This article has been retracted.

# Ecological Adaptability and Application of Traditional Historical Buildings under the Background of Environmental Protection

**DOI:** 10.1155/2022/5107325

**Published:** 2022-08-31

**Authors:** Min Yi, Wei Wu, Heng Su, Huiyuan Chen

**Affiliations:** He Xiangning College of Art and Design, ZhongKai University of Agriculture and Engineering, Guangzhou 510225, Guangdong Province, China

## Abstract

Traditional historical buildings carry the culture and spirit of China for thousands of years and have a unique charm that modern buildings do not have. However, traditional historical buildings have gradually declined over time, and their restoration not only takes time and materials but also causes certain harm to the environment. Therefore, this paper has aimed to explore how traditional historical buildings can develop in a sustainable and ecologically adaptive image in modern times. For traditional historical buildings, this paper has taken traditional cave dwellings in northern Shaanxi as an example to analyze their ecological adaptability, and based on the analysis results, traditional cave dwellings have been transformed. Specifically, this paper has taken the comfort of residential houses as the evaluation standard and has selected the thermal stability of the building and the energy consumption of heat supply as indicators to compare and analyze the traditional cave dwellings and the renovated cave dwellings. The experimental results of this paper have found that the traditional historical buildings are the crystallization of the wisdom of the ancients for thousands of years. However, due to the limitation of technology, the lighting and thermal stability of traditional cave dwellings are not high. After scientific design, the lighting and thermal stability of the transformed cave are 100% and 30% higher than those of the traditional cave, respectively, and the heating energy consumption is reduced by 50%.

## 1. Introduction

Traditional historical buildings have irreplaceable and nonrenewable value, and the wisdom, aesthetics, and creativity reflected in the construction process can inspire and further innovate the future village construction. Its ecological adaptability is also one of the key factors in the formation of traditional historical buildings and their continuous updating and adaptation to environmental changes. Traditional historical buildings have undergone more than a hundred years of evolution. The builders of each are based on the local environmental conditions, relying on their own understanding of space in a specific regional context, to create a unique order belonging to the local village, and gradually adapt to the environment and the integration of the environment to stimulate the potential of the environment itself. It is a typical case of ecological adaptive construction and has an extremely high research value. However, with the development of the economy, many villages have been blindly constructed, ignoring the regional characteristics. Lack of effective use of the local natural environment, the gradual patterning of village construction has caused damage to the environment and lost its unique form due to adaptation to the environment. It is hoped that through the research of this paper, the status quo of ecological adaptability of traditional historical buildings can be further understood and the advantages of ecological adaptability in the construction of traditional historical buildings can be compared. By comparing the advantages of ecological adaptability in the construction of traditional historical buildings, it provides a theoretical basis for the ecological adaptability construction of future villages in this area and solves the problems arising from village construction during the implementation of the rural revitalization strategy.

The formation of traditional historical buildings often takes decades or even centuries of accumulation, which contains the essence of traditional Chinese culture. There are many studies on the ecological adaptability of ancient villages. Xie has studied the ecological adaptation of Hani village landscape. He has mainly studied the reasons for the formation of rural landscape as a material carrier, the process of rural landscape adapting to nature and the built environment, and its inherent ecological significance from the perspective of ecological adaptability [1]. Shiyun Tang et al. has conducted on-the-spot analysis of traditional famous residences in many places in Guangxi, and has established different models for evaluation of the adaptability of traditional buildings [2]. Ramesh et al. has studied traditional dwellings on the Eastern Ghats of Andhra Pradesh, India, and it has assessed the ecological suitability of traditional dwellings [3]. The residences of Hani villagers are divided into 4 types: rammed earth house (earth palm house), mushroom house, tile house, and stilted house (dry barn house). Huang S. and Huang H. have analyzed the environmental adaptability of these buildings [4]. Heidrich et al. have put forward higher standards for the environmental adaptability of buildings and they have adopted stricter parameters to evaluate the environmental adaptability. Their research has contributed to the development of powerful tools for assessing building adaptability, which has enhanced the decision-making process for building design and the development of a more sustainable built environment [5]. However, their research goal is to maximize the preservation of ancient buildings and the environmental requirements are not very important.

Environmental protection is a necessary step for the sustainable development of human beings and the environmental protection of buildings is an important part of it. There are many scholars who have done research on green building and sustainable building. CSP Lopez has conducted an extensive, detailed, and accurate collection of case studies on the application of solar photovoltaic and thermal systems in historic buildings to assess the sustainability of historic buildings [6]. Greta et al. have developed a decision support system to plan and manage energy retrofit activities for cultural heritage. Cost and energy use were assessed, as well as the compatibility of interventions and their impact on indoor environmental quality [7]. Soyemi conducted research on the funds of the British Heritage Lottery Fund for the historical built environment, and he has proposed a new method of historical building conservation through the historical building conservation situation that has been funded [8]. Deggim et al. reconstructed the entire building, museum exhibits and six historical stages of construction based on the capture of 3D data [9]. Anisa and Lissimia aimed to describe the impact of the historic buildings in the Menara Kudus area on the sustainability of the surrounding area. They have analyzed field data using three dimensions of sustainability in the economic, social, and environmental domains [10]. However, most of their research objects are modern industrial buildings, and few scholars conduct research on the environmental protection and sustainability of historical and ancient buildings.

In this paper, the environmental adaptability and sustainable development of historical buildings have been studied. Without destroying the original environmental adaptability, the shortcomings of traditional historical buildings are improved by using modern technology, and finally, the sustainable development of traditional historical buildings is realized. It not only retains the cultural heritage of traditional historical buildings and the advantages of environmental protection but also improves the technical defects of traditional historical buildings. It has provided some help for the subsequent restoration and development of historical and ancient buildings.

## 2. Environmental Protection and Traditional Historical Buildings

### 2.1. Ecological Adaptability of Historical Buildings

Ancient villages refer to villages with a long history, most of which have existed for hundreds of years. At the beginning of the construction of the village, the population was often sparse, and after several years of reproduction, a huge family was gradually formed. Working people build their own homes on this land with their hard work and wisdom. The division of labor in ancient villages is clear, production and living are self-sufficient, and there is a strong sense of dependence on the ecological environment. Traditional historical buildings and their earthen buildings are examples of a high degree of integration with the environment. The traditional dwellings in the village are adapted to the climate and terrain and use the characteristics of local materials such as raw soil with strong heat storage capacity to maintain a relatively constant indoor temperature and ensure indoor comfort. It is a real low-carbon and environmentally friendly energy-saving building. The traditional historical buildings in various places are shown in Figure 1. After the reform and opening up, with the gradual emergence of public architectural works by international designers in various places, all kinds of buildings in China have followed the trend and converged. Buildings blindly focus on the appearance and volume, ignoring energy-saving needs and regional characteristics, resulting in the convergence of buildings in different places and the same urban appearance. China has rich cultural heritage and regional characteristics. This phenomenon of architectural style convergence has a destructive effect on the maintenance and development of Chinese architectural models. It not only causes waste of resources but also leads to the lack of traditional Chinese architectural culture. In the twentieth century, faced with the shortage of international resources and energy, the living environment is deteriorating. Contemporary architects realize the inferiority of abandoning regional characteristics and blindly following the trend, and turn their attention back to traditional dwellings that combine nature, environmental protection and energy saving, and adapt to local conditions. The traditional Chinese dwelling model, formed after hundreds of thousands of years of changes, is the result of the combined effect of the local ecological environment and regional culture [11].

In biology, ecological adaptation refers to “the ability of organisms to adapt to the ecological environment in which they live.” As the external environment changes, the creatures in nature will also change accordingly. This paper mainly studies the adaptability of traditional dwellings to the ecological environment. Specifically, it refers to the adaptive characteristics of the entire village and its courtyard dwellings to the ecological environment such as climate environment, topography, hydrogeology, etc. [12], as shown in Figure 2. Since adaptability to the natural environment is the first challenge that human settlements need to face in the early stage of formation, traditional historical buildings are typical in terms of ecological adaptability. The research on the construction of traditional historical buildings is also of great significance.

### 2.2. Sustainable Development of Buildings

Due to serious air pollution, environmental degradation, soil erosion, and other phenomena in recent years, people have begun to reflect on their own behavior. The theory of sustainable development arises from the contradiction between the overexploitation of resources and the limitation of resources, and it is the result of the development of human society. In 1987, the United Nations Commission on the World and the Environment formally proposed the concept of sustainable development, as shown in Figure 3, and defined it as “development that meets the needs of the present without compromising the ability of future generations to meet their needs” [13]. The birth of this concept has aroused the attention of governments and public opinion in various countries, and actively advocated the public to implement it in actual production activities. The concept of sustainability was first proposed by ecologists, who advocated a balance between the ecological environment and the degree of human exploitation of nature, and hoped to use environmental resources in a controlled manner. The United Nations Conference on Environment and Development in 1992 adopted a series of documents such as the Framework Convention on Climate Change and the Global Agenda 21, which clearly demanded that the environment should not be neglected while developing. “Sustainable development” is a wake-up call for countries and people all over the world and the trend is gradually infiltrating all fields.

In China, the construction industry is an important industrial pillar of the national economy. At present, China is in a period of vigorous urban construction, and the investment and energy consumption of buildings are also increasing year by year. In the planning and design of buildings, the model of consuming a lot of energy in exchange for immediate economic benefits should be abandoned, the ecological environment should be protected as much as possible, the emission of pollutants should be reduced, and a sustainable “ecological house” should be constructed according to local conditions [14, 15]. Today, China is unable to meet the high-load resource demand. Many cities have adopted staggered power consumption and fixed-point power rationing to alleviate the problems caused by resource shortages.

### 2.3. Thermal Stability of Buildings

Architecture first existed as a shelter to ensure human safety. With the emergence of settlements, the maturity of construction techniques and the expansion of building scale, safety requirements have become the lowest-level requirements of buildings. No matter how mature the construction technique is and how the theory of architecture develops, the safety and independence of the interior space from the influence of nature are always the most basic needs of architecture. Since it is hoped to create a suitable building space, correspondingly, it is hoped to maintain a stable indoor thermal environment under the changes of external factors, so that it can meet the requirements of use and the thermal comfort of the human body. In general, the principle of interference that affects indoor temperature is shown in Figure 4.

Solar radiation is weakened in the atmosphere when sunlight passes through the earth's atmosphere, the radiant heat of each spectral component is weakened to different degrees, but all satisfy the law of differential weakening. For light of wavelength *λ*, the law is expressed as follows:

(1) $$\begin{array}{c} {\text{dI}}_{\lambda }=I_{\lambda }\alpha_{\lambda }d_{x}. \end{array}$$

where *α*_*λ*_ is the radiative attenuation coefficient of light per unit thickness of the atmosphere.

After changing the formula, the thermal radiation flow and the distance from the sun to the ground are, respectively, integrated, and the integral weakening law of the single-frequency light in the spectrum is obtained [16].

(2) $$\begin{array}{c} f_{I_{0\lambda }}^{I_{t\lambda }}\frac{1}{I_{\lambda }}{\text{dI}}_{\lambda }=-f_{0}^{l}\alpha_{\lambda }d_{x}. \end{array}$$

Or it is written as follows:

(3) $$\begin{array}{c} I_{t\lambda }=I_{0\lambda }\exp\left(-{\bar{\alpha }}_{\lambda }l\right). \end{array}$$

In the formula, ${\bar{\alpha }}_{\lambda }$ is the integral value of *α*_*λ*_ within the integral limit.

For the entire wavelength range,

(4) $$\begin{array}{c} I_{m}=f_{0}^{\infty }I_{m\lambda }d_{\lambda }=f_{0}^{\infty }I_{0\lambda }p_{m\lambda }^{m}d_{\lambda }. \end{array}$$

Among them are the following equations:

(5) $$\begin{array}{c} m=\frac{l}{h}, \end{array}$$

(6) $$\begin{array}{c} p_{m\lambda }^{m}=\exp\left(-{\bar{\alpha }}_{\lambda }l\right). \end{array}$$

According to the mean value theorem of integrals, there must be *p*_*m*_^*m*^ that makes

(7) $$\begin{array}{c} I=p_{m}^{m}f_{0}^{\infty }I_{0\lambda }d_{\lambda }=I_{0}p_{m}^{m}. \end{array}$$

The formula is the commonly used attenuation law of the full spectrum.

The solar radiation received by a surface is divided into two parts, direct radiation and scattered radiation. The direct radiation and scattered radiation of the sun irradiate the ground and are reflected and then are reflected by the clouds, going back and forth many times, and the scattered radiation is greatly enhanced. Considering these three points, the total radiant intensity on any surface is obtained by deduction [17]:

(8) $$\begin{array}{c} I_{ma}^{T}=I_{m}\cos\;\theta +D_{mE}^{a}. \end{array}$$

In the formula, *θ* is the incident angle of sunlight on the surface and *D*_*mE*_^*a*^ is the total scattering intensity of the total scattered radiation from the sky and the ground on any surface.

The temperature radiation intensity of the black body surface is calculated by the following formula:

(9) $$\begin{array}{c} E=C_{0}{\left(\frac{T_{a}}{100}\right)}^{4}. \end{array}$$

The net radiative heat intensity (specific heat flow) released by the ground due to long-wave radiation is as follows:

(10) $$\begin{array}{c} q_{re}=C_{0}{\left(\frac{T_{a}}{100}\right)}^{4}-B_{r}C_{0}{\left(\frac{T_{a}}{100}\right)}^{4}=\left(1-B_{r}\right)C_{0}{\left(\frac{T_{a}}{100}\right)}^{4}. \end{array}$$

The annual and daily changes of air temperature are cyclical, because the solar radiation that causes this change in air temperature is cyclical. The temperature can be harmonically analyzed according to the change period according to the observation data of the meteorological station. It expresses the temperature as a Fourier series:

(11) $$\begin{array}{c} t_{e}=\bar{t}+\sum_{k-1}^{\infty }\Theta_{k}\cos_{k}\omega \left(\tau -\tau_{k}\right). \end{array}$$

In order to describe the thermal stability of the building, the abovementioned factors affecting the thermal stability of the building are combined, and the concept of outdoor comprehensive temperature is introduced. The comprehensive outdoor temperature is equivalent to an equivalent temperature, which takes into account the influence of outdoor air temperature and solar radiation, as well as the radiant heat effect of the interface between the envelope and the ground [18]. The outdoor comprehensive temperature is represented by *t*_*sa*_, and its calculation formula is as follows:

(12) $$\begin{array}{c} t_{sa}=t_{e}+\frac{p_{s}I}{a_{e}}-t_{1r}. \end{array}$$

When thermal insulation calculations are performed, the maximum value of the integrated temperature, the diurnal average, and its diurnal fluctuation amplitude must first be determined. The maximum comprehensive temperature is calculated as follows:

(13) $$\begin{array}{c} t_{sa,\max}={\bar{t}}_{sa}+At_{sa}. \end{array}$$

The average comprehensive temperature is calculated as follows:

(14) $$\begin{array}{c} {\bar{t}}_{sa}={\bar{t}}_{e}+\frac{p_{s}\bar{I}}{a_{e}}-t_{1r}. \end{array}$$

The amplitude of the day-night fluctuation of the integrated temperature is as follows:

(15) $$\begin{array}{c} At_{sa}=\left(A_{t_{e}}+A_{t_{s}}\right)\beta . \end{array}$$

The heat storage coefficient of the material refers to the ratio of the heat flow amplitude *A*_*q*_ on the surface directly receiving the thermal harmonic action to the temperature vibration radiation *A*_*θ*_ of this surface when the surface of one side of the envelope is subjected to thermal harmonics. The heat storage coefficient is represented by “*S*,” which is related to the material itself, and the unit is *W*/(*m*^2^ · *K*).

(16) $$\begin{array}{c} S=\frac{A_{q}}{A_{\theta }}=\sqrt{\frac{2\pi \lambda cp}{z}}. \end{array}$$

When the fluctuation period is 24 hours, then

(17) $$\begin{array}{c} S_{24}=0.51\sqrt{\lambda cp}. \end{array}$$

When the envelope structure is composed of composite multilayer materials, the thermal inertia index needs to sum up the thermal inertia index of each layer material, the method is as follows:

(18) $$\begin{array}{c} \sum D=R_{1}S_{1}+R_{2}S_{2}+\cdots +R_{n}S_{n}=D_{1}+\cdots +D_{n}. \end{array}$$

## 3. Ecological Adaptability of Traditional Buildings

Some ancient villages still retain the original ecological production workshops, which are rare and well-preserved ancient villages in the world, and the study of ancient villages is representative to a certain extent. This paper takes the adaptability factors of Shaanxi cave dwellings and the ecological environment as the point of convergence and reflects the importance of traditional dwelling protection by studying the influence and role of climate environment, topography, hydrogeology, and other aspects on traditional dwellings in Hougou [19]. This article can not only enhance the public's attention to traditional dwellings but also contribute to the dissemination of the essence of Chinese traditional culture, and then extract useful experiences that can be learned from the construction of contemporary villages and towns. The traditional cave dwellings studied in this paper are shown in Figure 5.

### 3.1. Adaptability of Building Materials

The thermal environment comfort in the building is not only related to the layout and construction of the house but also largely depends on the thermal performance of the building materials. Traditional dwellings on the Loess Plateau mostly use readily available natural materials such as soil, stone, wood, brick, and grass. The roof of the building is covered with blue tiles, which have strong heat storage properties and are conducive to thermal insulation. In the back ditch, adobe is often used as a maintenance wall. The 60 cm adobe wall and 30 cm outer bricks are commonly known as “gold-clad silver.” The entire space is wrapped with heavy materials to effectively reduce heat loss. Adobe, tile, and brick are thermally inert, conduct heat slowly, and take a long time for heat to pass through the material. When the sun shines on the roof and wall during the day, they absorb excess heat and store it in the material. When the temperature drops at night, the material transfers heat to the interior, thus playing the role of thermal insulation [20].

“Building materials reflect the nature of the materials used.” Stone, soil, and bricks are all readily available materials in ancient villages, so the common forms of cave dwellings include stone kilns, earthen kilns, and brick kilns. Hougou raw earth building adopts hoop kiln technique, clever use of loess resources, and easy-to-obtain materials to create a different architectural atmosphere. These materials are nonpolluting to the environment and can degrade naturally even if they are discarded after several years. In short, the use of local materials is conducive to energy conservation and environmental protection, and has a high degree of adaptability to the ecological environment. Buildings with different materials are shown in Figure 6.

### 3.2. Adaptability to Life

The underground drainage system of the ancient village is famous, which is amazing. In an ancient society where information was blocked and resources were limited, it was not easy for working people to build a complete drainage system. In terms of organizing drainage, the open ditch is combined with the dark channel. It starts from the highest point of the northern hillside of the village, passes through the village, and passes through the courtyard, forming two systems of Huanglong and Heilong, and finally flows through the drainage outlets in the southeast and southwest of the village into the Longmen River. The normal life of human beings is inseparable from the drainage system. Water is a resource that villagers rely on for their survival, especially for the Loess Plateau, which is arid, less rainy and has loose soil. Organized drainage is conducive to efficient use of water resources and avoidance of waste. However, it is not uncommon to see the phenomenon of cross-flow of sewage in some villages today, which is not seen in ancient villages. The Hougou, which has a history comparable to a modern drainage system, has a history of hundreds of years and it embodies the diligence and wisdom of the ancient villagers [21].

The relative height difference of the ancient village is 66 meters. The terrain fluctuates greatly, and the buildings are built on the cliff. This kind of terrain can easily cause soil erosion. If there is no reasonable drainage system, geological disasters such as landslides are prone to occur. The ancestors of the ancient village may have realized these conditions and built the drainage system of the ancient village. The main principle is as follows: rainwater flows down from the top of the highest level through the underpass and into the next level. After a certain distance, it flows into the lower-level waterway through the channel, until it flows into the lowest level and finally joins the Longmen River in front of the village. There is a drainage outlet at the southwest corner of the lowest depression in each courtyard, through which the drainage in the courtyard flows into the channel under the village road, and bluestone slabs or stones are laid on it. The canals connect every household, but people are not visible. This practice is like a sewer in a city. The drainage system of the ancient village stretches for kilometers, the tributaries and the main stream are scattered, and the canal trunks are connected to each other and eventually merge into the river. It not only helps to keep the village clean and tidy but also saves resources and avoids soil erosion.

### 3.3. Adaptability of Ventilation Methods

The ancients asked for the site to be “backed by the mountains and facing the water,” precisely considering the importance of “Tibetan wind.” There is a saying in ancient villages that “the wind will disperse,” so the wind is considered to be an important aspect of choosing a house. In fact, from a scientific point of view, wind is also a great threat to human health, so the idea of wind prevention is essential. When the cold wind strikes, the courtyard is the shield of the house and a windproof unit. The northwest wind prevails in the ancient village in winter. When building residential houses, try to avoid the buildings facing the northwest direction, and do not open doors and windows facing the northwest direction.

The back wall of the buildings in the ancient village compound is generally higher than the front eaves, and no windows are opened to the outside, so as to effectively resist the wind and sand. In order to avoid the biting northwest monsoon in winter, the gate of the house is generally located in the southeast corner or south of the courtyard. This layout is also conducive to the southeast monsoon blowing into the courtyard in summer, dispelling heat and dissipating heat and keeping the air fresh. Considering the existing layout of Hougou courtyard, when the northwest monsoon is raging in winter, people can hardly feel the wind in the courtyard, but they can hear the sound of howling wind outside the courtyard [22].

In addition to natural ventilation by heat pressure and wind pressure in a single building, most cave dwellings also use the self-circulation system formed by the flue, chimney, and cooking stove of the kang to enhance the ventilation effect. In this system, the stove mouth is at a relatively low position and belongs to the high pressure area and the chimney is at a relatively high position and belongs to the low pressure area. The flowing air will discharge the indoor foul air out of the cave through the chimney, keeping the indoor air fresh. In summer, the chimney is in the negative pressure area, and the power of natural ventilation is mainly the effect of wind pressure. In winter, the temperature of the stove mouth is high. At this time, natural ventilation mainly relies on the effect of heat pressure. The temperature difference between indoor and outdoor in summer and winter is large and the air pressure difference is obvious. The ventilation effect is better than that in spring and autumn.

## 4. Reconstruction and Application of Traditional Historical Buildings

### 4.1. Green Renovation of Ancient Village Cave Dwellings

Site selection and material selection is done according to local conditions.

Energy saving and environmental protection: here, the cave dwellings are built on the hillside. Through the stepped layout following the slope, the harmonious treatment of “integrating” into the environment is closely combined with nature. In addition, the caves built by using natural gullies will not damage the ecology or occupy fertile land, but also help to maintain water and soil resources and coordinate with the ecological environment. According to relevant information, “the cave dwelling is 20% more energy efficient than modern high-rise buildings.”

A livable environment with “warm in winter and cool in summer.”

Warm in winter and cool in summer, comfortable and practical. Traditional kiln dwellings are closed and regular, with concise planes, simple shapes, and relatively small shape coefficients, thereby reducing the impact of outdoor air temperature on the indoor thermal environment. The caves with thick loess and masonry as the enclosure structure are fireproof, noise-proof, and have good thermal insulation performance. Under the influence of large outdoor temperature fluctuations, the indoor temperature remains relatively stable.

The way of constructing “the unity of man and nature.”

Most of the traditional cave dwellings face south and are built on the hillside or the foot of the mountain. Most of the north faces are backed by mountains. According to the principle of mechanics, the construction is completed with a special arch structure, and the noise is low. The stove used for cooking in the cave is connected to the kang, and the smoke and waste heat generated by cooking are converted into radiant heat when passing through the flue, which transfers heat to the kang, and also meets the heating needs while cooking.

During the research period, in ancient villages, detailed tests and questionnaires were conducted on the old cave dwellings of Zhangjia Old Courtyard and the physical environment quality of residential areas.

The survey is divided into two parts: objective and subjective: the current situation of cave dwellings and the residents' intuitive feelings about cave dwellings. Among them, the main contents of the test and investigation include: indoor and outdoor thermal environment, light environment, acoustic environment, various harmful gases and dust in the air, thermal properties of cave building materials, outdoor climate and meteorological parameters, etc.

Indoor thermal environment: “warm in winter and cool in summer,” that is, the temperature is relatively stable throughout the year, as shown in Figure 7.

Acoustic environment: the sound field is uneven and there is sound focusing.

Light environment: the lighting coefficient is extremely uneven; air quality: poor ventilation and poor quality.

In order to create a more comfortable indoor thermal environment, the author conducted a field investigation and research on the Zhangjia Laoyuan, a representative Yuan Dynasty building in the ancient village. While fully affirming its construction technology, the aspects that affect the comfort of the occupants are reasonably transformed.

Cave dwellings usually use “one light and two dark,” several cave dwellings are connected in series with each other, and there are door openings inside.

The thick and heavy envelope of traditional cave dwellings is maintained. Due to the strong heat storage performance of loess and other materials, the interior is warm in winter and cool in summer, creating a comfortable and pleasant living environment.

Improvements are made by opening windows on the north side and setting up lighting and ventilation shafts. Using the principle of light reflection, setting mirror materials at appropriate positions in the shaft can effectively improve the lighting rate.

### 4.2. Application Strategies of Ecological Technology in New Residential Buildings in Contemporary Towns

In this paper, the cave dwellings, brick-wood structure dwellings with similar area and volume in the old courtyard of the old village of Zhangjia, and the newly built dwellings built by the descendants of the Zhang family outside the village are taken as the research objects, and their physical properties are analyzed through the calculation of heat consumption index and coal consumption:

It can be seen from Table 1 that the heat consumption index of newly built dwellings is significantly higher than that of traditional dwellings in cave dwellings and brick-wood structure dwellings, and the coal consumption is also much higher than that of traditional dwellings.

In addition, the thermal insulation and thermal insulation ability of the envelope structure is reflected in the barrier effect of the envelope structure on heat. The heat transfer resistance of the envelope structure is its blocking effect on heat, and its single material calculation formula is *R*=*d*/*λ*, as shown in Table 2:

After monitoring, without using any artificial equipment, the indoor temperature of traditional residential buildings in winter is 1.5–3°C higher than that of new residential buildings. The results show that in terms of indoor comfort, traditional dwellings are superior to newly built dwellings. New dwellings should inherit the advantages of energy saving of traditional dwellings, combine modern technology and materials, and build local buildings that are energy-saving and environmentally friendly. New residential buildings in villages and towns require the lowest possible energy consumption, and more attention should be paid to the ventilation and lighting of buildings, the recycling of energy and the selection of construction materials. In winter, it relies on its own materials to store heat and keep warm, and in summer, it is cooled by natural ventilation, and then integrates new technologies such as solar energy and geothermal energy to reduce living costs. Such houses must be talked about by villagers.

After several studies and determinations of the physical environment of the cave dwellings in the main house of the Zhangjia Old Courtyard, the author summarizes its suitability characteristics and the indicators that need to be renovated to affect the indoor comfort.

### 4.3. Thermal Stability and Energy Consumption

The reason why buildings generate energy consumption and follow its source is that people have different thermal needs in different environments. Buildings are based on a certain geographical environment. The building isolates the internal space from the external environment, but at the same time, the thermal environment of the internal space of the building is constantly affected by the external environment and internal conditions. The external environment is constantly changing, and the internal environment is affected by the common influence of various equipment and human body heat production. The indoor thermal environment is therefore constantly changing, while the human thermal demand is relatively constant. Due to these changes, the actual indoor thermal environment is different from the thermal environment expected by people to achieve comfort needs. In order to eliminate this difference, various ventilation, cooling, heating, dehumidification, and other equipment are used inside the building to adjust. For example, using central heating equipment to increase indoor air temperature in winter, reducing indoor air temperature through air conditioning equipment in summer, and dehumidifying equipment in places with high humidity are all means to eliminate differences.

The thermal comfort of the human body is related to six factors, and the factors related to the building itself are radiation temperature, air temperature, wind speed, and humidity. Through the device, the air temperature, wind speed, and humidity can be adjusted, but the radiation temperature cannot be controlled. To control the radiation temperature, the expected envelope temperature can only be controlled by designing the envelope structure, so as to achieve the purpose of controlling the radiation temperature. In desert areas, the moisture content is very low, and at the same time it is basically constant, the wind speed is not large, the sunshine is strong, the air temperature fluctuates greatly within 24 hours, and the comprehensive temperature of the building surface changes drastically under the combined effect. At this time, it is very important to select a suitable enclosure structure to resist the influence of the fluctuation of the comprehensive temperature on the indoor thermal environment, which is very important to maintain a stable indoor thermal environment.

How well the building is designed and how the building envelope is constructed is not only reflected in the numerical value but also needs to consider whether the human body feels comfortable in the building. Here, the neutral temperature calculated by the thermal comfort model in the dry-hot, dry-cold area is used to compare the operating temperature to evaluate whether the person feels comfortable in the room. The thermal comfort model represents the change of the comfortable temperature felt by the human body with the outdoor air temperature under certain climatic conditions. The thermal comfort model used in this paper is derived from the results of other members of the research group. The thermal comfort model of dry-hot and dry-cold regions can be expressed in the range of −10°C to 40°C.

(19) $$\begin{array}{c} y=0.019x^{2}-0.288x+18.25. \end{array}$$

*where x* is the outside air temperature and *y* is the neutral temperature.

The distribution of neutral temperature and operating temperature at each moment in summer and winter is shown in Figure 8.

It can be seen from Figure 8(a) that the operating temperature of the cavern will be higher than the neutral temperature from 13:00 to 23:00 at night, especially from 16:00 to 18:00, the difference is close to 2°C. However, it can still ensure that the thermal comfort needs of the human body can be met for most of the 24-hour period.

From Figure 8(b), it can be seen that the neutral temperature changes significantly with the outdoor air temperature, and the neutral temperature is the highest around 9 am in the morning. The neutral temperature is the lowest around 4:00 pm, which is also in line with the fact that the radiation intensity is not large in the morning when the sun just rises, and various functions of the human body are gradually adjusted from sleep. It is hoped that the higher indoor temperature is consistent with the common sense that the demand for indoor temperature begins to decrease in the afternoon with the enhancement of solar radiation and the deployment of human body functions to achieve the maximum effect.

In general, in winter, when openable components such as doors and windows are closed, the indoor operating temperature is quite constant, and the extremely low temperature outside has little effect on the indoor temperature. Especially under the heavy structure of the dwellings (caves), the influence of the extreme outdoor temperature within 24 hours can be ignored. Due to the good thermal stability of the envelope structure, the inner surface of the envelope structure is not greatly affected by the fluctuation of the outside temperature. Therefore, when adjusting the indoor thermal environment in winter, the indoor air temperature has become the only factor to be considered. At the same time, this factor is also easy to control through equipment or traditional stoves. It should also be noted that in the case of large amounts of solar radiation in the afternoon in winter, it is very beneficial to introduce solar radiation into the room reasonably to increase the indoor operating temperature, improve the comfort of people in the room, and save energy.

In summer, with natural ventilation, the operating temperature in the afternoon will be greater than the neutral temperature. At this time, closing the doors and windows to stop natural ventilation, preventing outdoor high-temperature air from entering the room, can effectively reduce the indoor operating temperature. At the same time, attention should also be paid to the surrounding environment of the building and the design of the shading components of the building itself. The former can reduce the amount of radiation directly received outdoors, thereby reducing the temperature of the air entering the room, while the latter can reduce a large amount of direct solar radiation entering the room and heat the air temperature in the room. It is precisely because of the good thermal stability of the envelope structure that the inner wall is less affected by fluctuations in outdoor temperature, making the control of indoor air temperature and wind speed the main consideration for improving the indoor thermal environment in summer.

In the calculation of this paper, the room heat transfer situation is idealized, and it is considered that the indoor air temperature in winter is constant and the structure is uniform, while the gaps, infiltration and thermal bridges existing in the actual building will affect the final indoor operating temperature results. The outdoor weather data used for the calculation are monthly averages, that is, the effects of extreme low temperatures are not considered. It is conceivable that when the temperature at night is extremely low, especially in weak parts such as windows, there is a cold radiation effect at night. In the absence of the thermal storage call cold radiation effect of the envelope, the radiant temperature of a room with a lightweight envelope can be significantly reduced. This means that a higher indoor temperature needs to be provided to increase the indoor operating temperature, and at the same time bring higher energy consumption. In addition, it can also be seen that in winter, the rational use of solar radiation is of great significance for room heating and reducing heating energy consumption.

For buildings with no natural ventilation and constant indoor air temperature, the effect of radiant temperature is more obvious. Figures 9(a) and 9(b) show the same thermal resistance, the attenuation factor of 60, the constant temperature room constituted by the envelope with the delay time of 5 hours and the attenuation factor of 10, respectively. A schematic diagram of the radiation temperature and operating temperature changes of the envelope with a delay time of 1 hour under the influence of the outdoor temperature harmonics is shown. Figures 9(a) and 9(b) show the same thermal resistance, the attenuation factor of 60, the constant temperature room constituted by the envelope with the delay time of 5 hours and the attenuation factor of 10, schematic diagram of the radiation temperature and operating temperature changes of the envelope with a delay time of 1 hour under the influence of the outdoor temperature harmonics, respectively. The outdoor meteorological parameters are still taken according to the local summer conditions. It can be seen that due to the selection of enclosure structures with different heat storage coefficients and structural forms, the attenuation factor differs by 6 times and the delay time differs by 5 times, resulting in a room with good thermal stability. The radiation temperature and operating temperature are very stable. In a room with poor thermal stability, although the air temperature is constant, the operating temperature still changes drastically under the influence of the radiation temperature change. That is to say, although the indoor air temperature is controlled within a constant range by means of equipment adjustment, if an inappropriate enclosure structure is adopted, the temperature felt by the human body will still change drastically. When the neutral temperature is distributed according to Figure 9(b), a larger cooling energy consumption is required to make a room with a small attenuation factor meet the comfort requirement. Due to the poor thermal stability, the radiation temperature of the room with a small attenuation factor changes drastically within 24 hours, resulting in the still drastic change of the operating temperature, which is very unfavorable in terms of energy saving and human physiological health.

### 4.4. Transformation Effect

In order to compare the advantages and disadvantages of the indoor environment quality of the kiln dwelling buildings before and after the renovation, a comprehensive simulation of the indoor thermal environment was carried out. Through comparison, an accurate evaluation can be made on the renovated cave dwelling buildings, which is of great significance to whether the new cave dwelling buildings can become a sustainable living model in the Loess Plateau. The thermal environment includes indoor and outdoor ambient temperature, daylighting coefficient, acoustic environment and acousto-optic environment, as shown in Figure 10, Tables 3– 5, respectively.

The abovementioned results show that the green-renovated cave dwelling not only inherits and retains its traditional advantages but also significantly improves the indoor comfort. The results show that the indoor physical environment quality of the renovated kiln house is better than that of the traditional kiln house. The new type of cave dwelling not only provides a good living model for the ancient villages on the Loess Plateau but also has substantial significance for the inheritance and extension of the local cultural context, and creatively improves the architectural living environment in the area.

Cave dwellings are products that conform to the natural ecology and social economy, and are the crystallization of the experience and wisdom of the working people. The green thinking contained in them makes them a typical example of energy saving and land saving. In contemporary architectural design, it is necessary to learn from the experience of ecological architecture embodied in traditional dwellings, and to develop it according to the characteristics of the times. Especially in the design process of residential buildings in local towns, it is necessary to be good at using ecological language to make residential buildings more livable.

## 5. Conclusions

With the rapid development of the global economy and the accelerating process of urbanization, countless high-rise buildings across the country have been erected, resulting in more and more traditional dwellings disappearing from people's sight. While blindly pursuing immediate interests and comforts, the environment has also given human beings a blow. Climate deterioration, resource depletion, soil erosion and other problems that have appeared in recent years are all caused by human overdevelopment in violation of the laws of nature. Traditional ancient villages and their dwellings are living models that are compatible with the ecological environment and are the result of sustainable development. Studying the ecological strategies for their construction has a good reference value for contemporary village construction and architectural design. The disadvantage of this paper is that the relevant calculations and software simulation operations are carried out under ideal conditions and the results are inevitably slightly biased. The authors used meteorological data from the nearest area, but can guarantee that the final result will not be affected. Therefore, in the follow-up research, more historical and traditional buildings and more ancient villages will be studied.

## Figures and Tables

**Figure 1:** Traditional buildings with different styles.

**Figure 2:** Ecological environment adaptability.

**Figure 3:** Sustainability.

**Figure 4:** Building indoor and outdoor environmental interference.

**Figure 5:** The real picture of traditional cave architecture. (a) Cave house. (b) Cave room. (c) Cave house door.

**Figure 6:** Buildings with different materials. (a) Soil. (b) Stone. (c) Wood.

**Figure 7:** Indoor thermal environment of the cave. (a) Indoor and outdoor temperature comparison in summer. (b) Indoor and outdoor temperature comparison in winter.

**Figure 8:** Comparison of neutral temperature and operating temperature. (a) Summer neutral temperature and operating temperature distribution. (b) Winter neutral temperature and operating temperature distribution.

**Figure 9:** Effects of different attenuation factors on operating temperature and radiation temperature. (a) Radiation temperature comparison at different attenuation times. (b) Operating temperature comparison at different attenuation times.

**Figure 10:** Comparison of indoor temperature before and after renovation. (a) Comparison of indoor temperature in winter before and after renovation. (b) Comparison of indoor temperature in summer before and after renovation.

**Table 1:** Differences between traditional buildings and new residential buildings.

		Wall thickness (cm)	Window to wall ratio	Body shape factor	Heat consumption index (W/m^3^)	Coal consumption for heating (t)
*Traditional building*	Cave	100	0.12	0.35	18	1
	Brick and wood structure dwellings	50	0.18	0.50	20	1.2
Newly built dwellings		40	0.37	0.55	22	2

**Table 2:** Calculation of thermal resistance of the wall.

	Rammed clay	Grassed clay	Brick
*λ*[*W*/(*m* · *K*)]	1.32	0.78	0.82
*d* (m)	0.88	0.43	0.38
*R*	0.67	0.55	0.46

**Table 3:** Daylighting coefficients before and after renovation.

Distance from the window (m)	Transformation of the former (%)	After transformation (%)
0	17.3	31.5
3	3.6	10.6
6	1.4	1.9
9	0.4	0.4

**Table 4:** Cave acoustic environment.

	Transformation of the former	After transformation
Background noise (dB)	27.3∼30.2	27.3∼29.4
Noise when no one speaks (dB)	24.3∼31.8	33.3∼39.5
Noise when someone is talking (dB)	24.1∼54.5	43.2∼53.1

**Table 5:** Cave light environment.

	Outdoor (lx)	Indoor (lx)
Suitable light intensity	—	1000
Transformation of the former	40500	400
After transformation	40500	1100

## Data Availability

The data that support the findings of this study are available from the corresponding author upon reasonable request.
